This article has been retracted.

# Implicit Environmental Injustice in Global Trade: Based on the MRIO Model

**DOI:** 10.1155/2022/7520510

**Published:** 2022-08-11

**Authors:** Ping Zhang, Tianjiao Zhang, Ranran Meng, Shiwen Jiao

**Affiliations:** ^1^School of Marxism, Xinxiang Medical University, Xinxiang 453003, Henan, China; ^2^School of Economics, Party School of the Central Commmittee of CPC (National Academy of Governance), Beijing 100091, China; ^3^School of Economics, Shanghai University, Shanghai 200444, China; ^4^School of Business, Henan Normal University, Xinxiang 453002, Henan, China

## Abstract

To answer these questions in light of the MRIO model, this paper presents a study of environmental injustice affecting the global economy. Practical ideas and lifespan measurements are often used in studies of the embodied carbon industry. The input-output table method is an important method for industrial embodied carbon research, which can be divided into the regional input-output table method, bilateral input-output table method, and multiregional input-output table method. Bilateral and multistakeholder consultations are more accurate than regional proposals. Therefore, when studying the carbon industry implied by the two countries, the input-output table of the two countries is usually used, and the multilateral input-output table is more reliable for determining the input-output calculation. Therefore, when studying local problems, it is advisable to adopt a variety of display strategies. The results show that in 2010, the carbon content of the carbon industry was 26,593 thousand tons, down 34.6% from 17,383 thousand tons in 2011, calculated at 2%. From 2012 to 2018, the carbon content grew from 31,051 tons in 2014 to 84,248 tons in 2018, with an average annual increase rate of 18%. The experimental results show that there is a large incidence of carbon emissions in the bilateral trade between China, the United States, and Japan. The expansion of export industries is the main reason for the increase in carbon emissions between the two industries. The role of technology has narrowed this difference to some extent.

## 1. Introduction

Our business revolution has had a profound impact on facilitating international trade and technological progress. However, since the industrial revolution, especially the first two economic revolutions, developed countries have also brought many environmental problems in the process of increasing the achievements of the industrial revolution. The global climate is slowly warming, the ecological environment is slowly deteriorating, and the living environment is declining. The successful development of industrialization is an incomplete result of the industrial revolution. Of course, a series of developments have also brought a series of environmental problems and environmental crises. Since the reform and opening up, China's participation in international trade has gradually been criticized, although all import and export packaging of China once surpassed the United States to become the world's largest exporter. However, in the process of continuous improvement of the industry, the environmental injustice behind it is very obvious. After all, China often runs a surplus in international trade. Coupled with incomparable international economic standards, lack of energy, and low energy consumption, China is the main exporter of implied carbon emissions in the international market, which undoubtedly increases the pressure on foreign markets to reduce emissions. Therefore, this paper provides an in-depth study of climate change and the environmental injustice implicit in the Chinese economy based on the MRIO model, as shown in Figure 1.

## 2. Literature Review

The most important research studies currently focus on emissions accounting and the distributional role of production and consumption, carbon emissions accounting and virtual exchange fields or domestic industries under the influence of globalization, pollution caused by industries, losses affecting the environment and health, thinking and prosperity, affecting environmental injustice, and so on. In the context of global trade integration, commercial pollution in some countries will transfer pollution-intensive industries to nonpolluting countries and regions, and there are few environmental laws and principles, that is, the “Rock Slab Hypothesis.” Heavy electrical equipment is still being exported to food-producing countries. This also creates the problem of implicit pollution in the country or region. Especially in terms of greenhouse gas emission reduction, because the Kyoto Protocol does not specify the greenhouse gas emission reduction targets of developing countries, it is creating countries to transform carbon emission-intensive industries into developing countries (such as China and India). Although greenhouse gas emissions have decreased, it is possible to increase carbon emissions because developed countries have higher carbon emissions than developed countries. Emissions on earth are increasing. To achieve global greenhouse gas emissions is extremely difficult. Scientists call this phenomenon carbon leakage.

Entering the 21st century, some scientists began to analyze the details of the final product on a design basis and the use of end-to-end emissions accounting and financial processes to determine the role of final production and final emissions from a design perspective. Balance and analyze the content of the final product and final emissions allocation and assignment responsibility. Through statistics, the transfer of developed countries to industrialized countries is determined, which proves the problem of “carbon to” globalization and points out that in the post-Tokyo Protocol era, it should be decided to calculate the national emission status. Currently, consumer-based accounting is widely used around the world and integrates carbon monoxide, equipment, land use, water use, pollution, healthy environment, and more. It has been proved from multiple perspectives that developing countries or regions that use less heavy metals and pollutants consume more energy and resources and emit more pollutants [1].

In recent years, some researchers have paid particular attention to the carbon impact of industries such as agriculture. Some scientists have studied carbon monoxide in the foreign trade of my country's agricultural products in 2002 from the perspective of a single industry and found that my country's agricultural products still have carbon sink problems. As far as agricultural products are concerned, China's main exporter of carbon is Asia, while North America, Latin America, and Asia are the main exporters; this paper explores carbon emissions from U.S. agricultural products and examines carbon emissions across life from a food perspective. The results show that for agricultural products that need to be transported for a long time, the CO_2_ emissions generated during the production phase account for 83% of the entire life cycle; through the analysis of the carbon footprint, this paper explores different horticultural products in Germany and artefacts from other countries and analyzes many carbon emissions in the life cycle of various products which were compared horizontally. The study found that the carbon footprint of horticultural products varies widely, with consumption-level GHG emissions ranging from 3% to 71% of total life-cycle emissions, while horticultural materials contribute to GHG emissions from fertilizer use. The phase is very large [2].

## 3. Model Construction of Implicit Environmental Pollution Based on International Trade

### 3.1. Construction of the Multiregional Input-Output Model

In the competitive input-output model, the state relationship is shown in

(1) $$\begin{array}{c} \sum_{j=1}^{n}a_{ij}X_{j}+y_{i}=X_{i},\;i=1,2,\ldots ,n, \end{array}$$

where is the output of cell *j*, which must take input directly from cell *i*, which is derived from sheet/*X*_*j*_. *Y*_*i*_ represents the final demand of office *i*, and *X*_*i*_ is the total product of office *i*. Multiple regional input-output models can be extended based on a country's noncompetitive input-output table. The basic models of various regional input-output models are shown in Table 1.

Assuming that there are *n* countries or regions in the world, the MRIO model can be expressed as shown in

(2) $$\begin{array}{c} \left(\begin{array}{c} X^{A}\\ ...\\ X^{N} \end{array}\right)=\left(\begin{array}{c} \begin{array}{ccc} A^{AA} & ... & A^{AN} \end{array}\\ \begin{array}{ccc} ... & ... & ... \end{array}\\ \begin{array}{ccc} A^{NA} & ... & A^{NN} \end{array} \end{array}\right)\left(\begin{array}{c} X^{A}\\ ...\\ X^{N} \end{array}\right)+\left(\begin{array}{c} Y^{A}\\ ...\\ Y^{N} \end{array}\right). \end{array}$$

The vector to the left of the symbolic equation in the above model is the sum of all values for each sector in country *Q*, corresponding to the last row of all outputs in Table 1. On the right side of the equation board is the matrix *A*, the direct supply matrix, which represents the direct input of one country and the quantity consumed by each factor in the other country. A house in country *Q* is a unit of output. This provision is the same as above. The second product on the right-hand side of the symbolic equation is the total product of the sectors of country *Q*. The last vector on the right-hand side of the equation is the final application of country *Q* to the product of itself and other countries, which can be decomposed into

(3) $$\begin{array}{c} \left(\begin{array}{c} Y^{A}\\ ...\\ Y^{N} \end{array}\right)=\left(\begin{array}{c} y^{AA}+\sum_{Q\neq A}y^{AQ}\\ \begin{array}{cc} \; & ... \end{array}\\ y^{NN}+\sum_{Q\neq N}y^{NQ} \end{array}\right). \end{array}$$

When *Q* ＝ *S*, *y*^*QS*^ represents the products directly used for end use provided by country *Q* to its own country. When *Q* ≠ *S*, *y*^*QS*^ represents the products directly used for end use provided by country *Q* to other countries.

Combined with formulas (1) and (2), the multiregional input-output model can not only reflect the input-output relationship between domestic departments but also reflect the input-output relationship between regional departments. The intermediate input matrix (from the column view) describes the input structure of domestic products in various sectors and products imported from other countries. The direction describes the specific use of products in each sector in their own countries and other countries.

The matrix of formula (4) is as follows:

(4) $$\begin{array}{c} X=AX+Y. \end{array}$$

After finishing, it can be obtained as shown in

(5) $$\begin{array}{c} \left(I-A\right)X=Y. \end{array}$$

The Leontief inverse matrix is as shown in

(6) $$\begin{array}{c} L={\left(I-A\right)}^{-1}, \end{array}$$

where *I* is the identity matrix, formula (7) can be expressed as

(7) $$\begin{array}{c} X=LY. \end{array}$$

We can use the MRIO model to describe the “climate change” of a region. Since each unit has a different level of technology, *E*^*Q*^ is a linear vector resulting from direct radiation, as shown in

(8) $$\begin{array}{c} E^{Q}=\left(\begin{array}{c} e_{1}^{Q}\\ e_{2}^{Q}\\ ...\\ e_{n}^{Q} \end{array}\right). \end{array}$$

The global direct emission coefficient vector is *e*, as shown in

(9) $$\begin{array}{c} E=\left(E^{A^{\prime }},E^{B^{\prime }},...,E^{N^{\prime }}\right). \end{array}$$

Referring to the complete consumption coefficient proposed by Leontief, the global pollution complete emission coefficient *E*_*p*_ can be further constructed, which is given by the following formula, as shown in

(10) $$\begin{array}{c} E_{p}=E{\left(I-A\right)}^{-1}=EL, \end{array}$$

where the complete emission coefficient of country *Q* is *E*_*p*_^*Q*^, and the final output matrix of country *Q* is shown in

(11) $$\begin{array}{c} Y^{Q}=\left(y^{QA},y^{QB},\ldots ,y^{QQ},\ldots ,y^{QN}\right). \end{array}$$

Thus, the pollution emission matrix of national *Q* based on production end accounting can be obtained, as shown in

(12) $$\begin{array}{c} PO^{Q}={\overset{⌢}{E}}_{p}^{Q}Y^{Q}, \end{array}$$

where ${\overset{⌢}{E}}_{p}^{Q}$ is a diagonal matrix whose diagonal elements are the corresponding elements in *E*_*p*_^*Q*^, and other nondiagonal elements are zero. The final demand column vector of region *Q* is as shown in

(13) $$\begin{array}{c} D^{Q}={\left(y^{AQ},y^{BQ},\ldots ,y^{QQ},\ldots ,y^{NQ}\right)}^{\prime }. \end{array}$$

Then, the pollution emission matrix based on consumer accounting in region Q is as follows, as shown in

(14) $$\begin{array}{c} DO^{Q}={\overset{⌢}{E}}_{p}D^{Q}, \end{array}$$

where ${\overset{⌢}{E}}_{p}$ is the diagonal matrix in which the diagonal element is the corresponding element of the corresponding row in *E*_*p*_, and the other nondiagonal elements are zero. Therefore, the pollution emissions at the production end and consumption end of region *Q* can be calculated, respectively, according to the above two formulas, as shown in formulas (15) and (16).

(15) $$\begin{array}{c} \text{Pollution discharge from production end of region }Q=\sum_{i=1}^{n}PO_{i}^{Q}, \end{array}$$

(16) $$\begin{array}{c} \text{Region }Q\text{ consumption pollution emissions}=\sum_{i=1}^{n}DO_{i}^{Q}. \end{array}$$

The research is primarily based on studies of the environmental impact of China and its industries. Therefore, more regional input-output models including China and its trading partners need to be developed. Based on the characteristics of the Chinese economy, we divide Chinese business partners into five regions: EU, Japan, US, rest of Asia, and rest of the world. Therefore, this paper will create multiple regional input-output tables for six regions and multiple industries [3].

### 3.2. Data Processing

Business integration. The standard input-output table provided by WIOD data divides the industry into 35 regions, international business models, while business information is divided into transportation, industry, and so on. To put the data together, we have broken down 8 sectors by industry in terms of inputs. We distribute UNCTAD's products to multiple industries, and industry services select trade data from the UNCTAD database [4] (see Table 2 for details).

Regional integration. The first data provided by the World Input-Output Database (WIODD) is a multicountry conference with 35 stores in 46 countries and a total of 1618 × 1841 matrices. After the joint venture, we added 46 regions to form a regional consensus. The benefits of division are as follows: (1) European Union: 28 member states, including Austria, Belgium, Germany, France, Italy, and the United Kingdom. (2) Asian Holidays: Korea, Malaysia, the Philippines, Thailand, Vietnam, Indonesia, India, Turkey, Russia, and Chinese Taipei. (3) Japan (4) United States (5) China (6) Other World: not all countries (or regions) above. Due to the wide range of data and matrix functions, most of the research was performed on data matrices and matrix counts via the MATLABsoftware [5].

## 4. Current Situation of China ASEAN Trade

### 4.1. Current Situation of Import and Export Trade between China and ASEAN

The entire trade bloc between China and ASEAN is developing rapidly. As can be seen from Figure 2, the export volume and import volume between China and ASEAN has increased from US$14.3 billion in 2010 to US$514.8 billion in 2020, an increase of 36 times [6].

There are approximately four stages of development and two stages of decline in this process. The first growth phase was from 2010 to 2012. In the past two years, the bilateral trade volume between China and ASEAN has grown steadily from US$14.3 billion to US$39.5 billion. From 2012 to 2014, sales increased by $252, experiencing a growth rate of 176% and an average annual growth rate of 16%. The second growth phase was from 2014 to 2016, and this phase grew rapidly, from $41.6 billion in 2018 to $231.3 billion in 2020. In 10 years, it increased by 189.7 billion US dollars, an increase of 456%. The average annual growth rate is 27% [7].

Before 2010, China's three major markets were the European Union, the United States, and Japan. However, since 2010, ASEAN has surpassed Japan to become China's third-largest economy, after the European Union and the United States.  Figure 3 shows the shift of key players in China. As can be seen from the figure, the bilateral trade between ASEAN and China is increasing year by year, and the gap with the EU and the United States is getting smaller and smaller. In the next few years, it may also catch up with the United States and the European Union to become China's largest economy [8].

In 2010, the total bilateral trade between China and ASEAN only accounted for 6.06% of China's total foreign trade. In that year, Japan's share was 20.25%, the US's share was 14.94%, and the EU's share was 18.51%. However, by 2017, ASEAN integration had shifted to 12.54%. In contrast, Japan's share is only 7.38%, and the US and EU's shares remain unchanged at 14.22% and 18.42%, respectively [9].

From 2012 to 2014 after the subprime mortgage exit, the packaging industry in China and the United States declined, and the industry share declined accordingly, but it recovered to more than 14% in 2016. ASEAN's share of China's foreign investment in trade volume increased almost every year. Only in the years severely affected by the financial crisis, the growth rate has been flat or slightly lower. However, as an important trading partner of China, ASEAN has become an important factor in the development of China's foreign trade [10].

Figure 4 shows the distribution of China's exports to ASEAN in China's total exports. It can also be seen from the figure that in 2017, China's exports to ASEAN reached US$279.120 billion, accounting for 12.33% of China's total exports that year. Compared with 2010, the total export volume between China and ASEAN was US$71.6055 trillion, accounting for only 5.92% of the total export value in that year. In eight years, exports have grown nearly 39 times. In addition to the decline in China's exports to ASEAN in 2010 due to the East Asian financial crisis and US subprime borrowing in 2011, China's packaging exports to ASEAN have also increased year by year. ASEAN is undoubtedly an important trading partner of China. It is of great significance to study carbon emissions in bilateral trade between China and ASEAN [11, 12].

### 4.2. Analysis of Trade Volume between China and Six ASEAN Countries

Although the China-ASEAN Free Trade Area is a joint venture project between China and the ten ASEAN countries, the trade volume between China and the ten ASEAN countries is different. As can be seen from Figure 5, the average trade volume between China and ASEAN countries from 2010 to 2017 was 16% in Brunei, 25% in Myanmar, 48% in Cambodia, and 11% in Laos [13, 14].

It can be seen that among the ten ASEAN countries, China's main markets are Brunei, Myanmar, Cambodia, and Laos. Since the calculation requires data input from ASEAN countries, but there is no data separation for Brunei, Laos, Myanmar, and Cambodia data, the ten ASEAN countries are divided into ASEAN countries and four ASEAN countries, respectively. The six ASEAN countries are Singapore, Malaysia, Thailand, Vietnam, Indonesia, and the Philippines. The other four ASEAN countries are Cambodia, Brunei Darussalam, Laos, and Myanmar. Since the trade area between ASEAN and other countries is added to Figure 6, the trade balance between ASEAN and China will be moved to Figure 6, which will also affect the accuracy of Figure 6.

It can be seen that the total bilateral trade between the four ASEAN countries and China has been less than 5% over the years, reaching 7.68% in 2014 and 5.35% in 2015. From 2010 to 2020, these countries accounted for 96.5% of the whole packaging industry between ASEAN and China [15]. Therefore, in the following two-sided market embodied carbon calculation, this paper selects Malaysia, Singapore, Thailand, Vietnam, Indonesia, and the Philippines as the representatives of ASEAN, while the other countries Myanmar, Laos, Brunei, and Cambodia are cancelled.

## 5. ASEAN China Trade Implied Perspective

### 5.1. Analysis of Total Implied Carbon in Bilateral Trade

This paper uses Eora subenergy sector data and YUN-GIO input-output series data to calculate CO2 emissions in China and ASEAN.  Figure 7 shows China and ASEAN's total CO_2_ imports, exports, and net exports in kilotons (Kt). It can be seen that, except for the decline in carbon emissions from China's exports in 2011 due to the global financial crisis in 2010, China's carbon monoxide exports to ASEAN have maintained a rapid growth [16].

As mentioned earlier, due to the impact of the East Asian economic crisis, trade between China and ASEAN remained stable and rebounded slightly in 2010. Therefore, from 2010 to 2021, the carbon emission exchange rate of China's exports to ASEAN is also very stable. In 2010, the hidden content of the carbon industry was 26,593 thousand tons, which dropped to 17,383 thousand tons in 2011, a decrease of 34.6% and then increased slightly in the following three years, increasing by 5.6%, 31.5%, and 2%, respectively. From 2012 to 2018, it grew rapidly, from 31,051 thousand tons in 2014 to 84,248 thousand tons in 2018, with a growth rate of 171% and an average annual growth rate of 18% [17].

### 5.2. Country Analysis of Implied Carbon in Bilateral Trade

As mentioned earlier, the economic relationship between China and ASEAN countries is not the same. In China's economic relationship with ASEAN, Malaysia, Singapore, and Thailand are more important. Therefore, it is necessary to verify the import and export of carbon dioxide in China and some ASEAN countries.  Figure 8 is a map of carbon country areas analyzed for China's exports to ASEAN, showing the integration of Singapore, Malaysia, Thailand, Indonesia, the Philippines, and Vietnam in China's exports to ASEAN in embodied carbon [18]. As can be seen from the graph, Chinese exports to Singapore, Thailand, Indonesia, and Vietnam have a greater impact on carbon emissions. Malaysia and the Philippines have relatively small carbon emissions and are managed equally [19]. From 2010 to 2022, China's carbon monoxide exports to ASEAN countries will be on par with other countries. In subsequent years, CO_2_ exports to Singapore and Indonesia have been the share of other countries, while Vietnam has gradually increased from 2011 to the same proportion as Malaysia and Singapore, and the other countries have remained mostly unchanged.

Figure 9 is the area chart of country analysis of carbon content in trade imported from China to ASEAN. What we want to explain here is that the first and second industries are excluded from the calculation of import implied carbon of Singapore because most of the data of these two industries in Singapore are zero, and their total carbon dioxide emissions are less than 1000 kilotons. For convenience of calculation, 29 industry matrices are used to calculate separately for Singapore. It can be seen that the implied carbon emissions imported by China from ASEAN mainly come from Thailand, Malaysia, and Indonesia, and Singapore and the Philippines account for a small proportion. However, the implied carbon emissions imported from Vietnam have risen rapidly since 2011 and exceeded the implied carbon imported from Indonesia in 2013. It can be seen that Thailand, Indonesia, and Vietnam are countries with a relatively high proportion of China's export and import implied carbon emissions, but Singapore has a small import volume despite China's export implied carbon. On the contrary, Malaysia has a small export proportion but a high import proportion [20].

Figure 10 shows the trade implied carbon of China's net exports to ASEAN countries. It can be seen that the trade implied carbon emissions of China's imports from ASEAN countries are lower than those of China's exports to six ASEAN countries, and the net exports of implied carbon are positive. Singapore and Indonesia are the two countries with the highest implied net carbon exports in China, and the implied net carbon exports show an upward trend. In 2010, the implied carbon emissions of China's net exports to Singapore were only 5000 kilotons, but by 2022, the implied carbon emissions of net exports had reached 30962 kilotons, an increase of 519%. The implied carbon net exported to Indonesia reached 22939 kilotons in 2022, an increase of 380% compared with 4775 kilotons in 2020 [21].

### 5.3. Analysis of the Implied Carbon Industry in Bilateral Trade

According to the industry classification standard of Eora database and the 35 industries defined in ISIC Rev 3.0 industry classification and YUN-GIO, this paper finally determines the classification details of 9 industries used in the calculation of the multiregional input-output table. At the same time, in order to facilitate industry analysis, the industries are further summarized into 5 categories. They are listed in Tables 3 and 4 [22].

Figure 11 shows the top eight industries with the largest export implied carbon emissions after calculating the implied carbon emissions of 31 industries from 2010 to 2020. These eightindustries are mining and quarrying, water and electricity supply, transportation, chemical and pharmaceutical industry, construction industry, petroleum refining industry, agriculture, forestry, animal husbandry, fishery, and base metals. Among them, the implied carbon export emissions of quarrying and mining and water and electricity supply are the most, accounting for almost 50%. Agriculture, forestry, animal husbandry, and fishery also accounted for more than 10% before 2011, but the share decreased in the following years and increased to more than 10% again in 2012. From 2010 to 2014, the quarrying and mining industry accounted for more than 30% of the exports of the top eight industries, but it fell sharply to about 10% in 2012, and other industries remained basically stable [23]. From the perspective of the growth rate, the industries with the fastest growth rate of China's implied carbon emission exports from 2010 to 2020 are communication equipment, electrical and mechanical equipment, other transportation equipment, medical and social services, and automobile manufacturing, with growth rates of 884%, 735%, 999%, 914%, and 1609%, respectively.

Figure 12 shows the export of implied carbon emissions of China's three major industries. It can be seen that primary and natural resources have always been the industry with the largest proportion of implied carbon emissions in China's trade exported to ASEAN. By 2010, almost all showed an upward trend, and they are much higher than the other four industries. Since 2011, the export implied carbon emissions of primary and natural resource industries have decreased, which was the same as that of the energy industry and heavy industry in 2011. In 2012, it was caught up by the energy industry, service industry, and heavy industry but still maintained high export implied carbon emissions.

Figure 13 shows the distribution of China's three industries importing implied carbon from ASEAN. It can be seen that the energy industry has always been the industry with the largest amount of implied carbon imported by China. From 2010 to 2020, it showed a rapid growth mode, rising from 3358 kilotons in 2010 to 13387 kilotons in 2011, an increase of almost four times. Different from the primary and natural resource industries, which are the most exported industries in China, the primary and natural resource industries are the industries with the least implied carbon imported by China from ASEAN. They have been maintained at the level of less than 2000 kilotons for 10 years and only increased in 2012, surpassing the original light industry in the last two places. The growth trend of implied carbon imports of the light industry, service industry, and heavy industry is similar, showing an upward trend from 2010 to 2022. Among them, the heavy industry has increased from 851 kilotons in 2010 to 8301 kilotons in 2020, an increase of nearly 10 times.

## 6. Conclusion

From the above data analysis, it can be seen that in the bilateral trade between China and ASEAN, China's economic embodied carbon emission exports are greater than China's economic and trade embodied carbon imports. From 2010 to 2022, China's embodied carbon emission exports also increased significantly. Net industrial means carbon exports have grown by more than 700% in 10 years. In fact, China plays a big role in ASEAN's carbon emission responsibility. From a country perspective, the embodied carbon trade between China and ASEAN countries also shows the status of China's net exports of embodied carbon throughout the year. The largest embodied carbon emissions from Chinese exports go to Singapore and Indonesia. Most of the embodied carbon imported from ASEAN comes from Malaysia and Thailand. Singapore exports very little carbon to China, and the carbon imbalance is even worse in Singapore.

In terms of industry, China's largest exports to ASEAN are primary and natural resource industries, and the heavy industry has grown the fastest, but the implied carbon emissions of imports are relatively low, and the volume of energy trade is relatively large, imported from China by ASEAN. In recent years, the import and export of the heavy industry, light industry, and light industry have increased, and bilateral trade between these industries has also been active, which further indicates that China and ASEAN have similar economic models, integrated and competitive trade.

## Figures and Tables

**Figure 1:** Based on the MRIO model.

**Figure 2:** China—ASEAN bilateral trade volume.

**Figure 3:** Proportion of total bilateral trade of major trading partner countries.

**Figure 4:** Proportion of China's exports to ASEAN in China's total exports.

**Figure 5:** Average trade volume between China and ASEAN countries from 2010 to 2017.

**Figure 6:** Total bilateral trade between China and ASEAN.

**Figure 7:** Implied carbon import and export volume of China—ASEAN trade.

**Figure 8:** China's exports of trade implied carbon emissions by country (1).

**Figure 9:** China's imports of trade implied carbon emissions by country (2).

**Figure 10:** Implied net carbon exports of China's trade.

**Figure 11:** Implied carbon emissions of China's export trade by industry.

**Figure 12:** Implied carbon emissions from exports of China's three major industries.

**Figure 13:** Implied carbon imports of China's three major industries.

**Table 1:** Multiregional input-output model.

Intermediate use										End use			
Intermediate input	Region *A*			…	Region *N*			Region *A*	…	Region *N*	Total output
	Region *A*	1	…	*n*	…	1	…					*n*
		1	*X *_11_^*AA*^	…	*X *_1*n*_^*AA*^	…	*X *_11_^*AN*^	…	*X *_1*n*_^*AN*^	*y *_1_^*AA*^	…	*y *_1_^*AN*^	*X *_1_^*A*^
		…	…	…	…	…	…	…	…	…	…	…	…
		*n*	*X *_*n*1_^*AA*^	…	*X *_*nn*_^*AA*^	…	*X *_*n*1_^*AN*^	…	*X *_*nn*_^*AN*^	*y *_*n*_^*AA*^	…	*y *_*n*_^*AN*^	*X *_*n*_^*A*^
	…	…	…	…	…	…	…	…	…	…	…	…	…
	Region *N*	1	*X *_11_^*NA*^	…	*X *_*nn*_^*NA*^	…	*X *_11_^*NN*^	…	X_1*n*_^*NN*^	*Y *_1_^*NA*^	…	*Y *_1_^*NN*^	*X *_1_^*N*^
		…	…	…	…	…	…	…	…	…	…	…	…
		*n*	*X *_n1_^*NA*^	…	*X *_*nn*_^*NA*^	…	*X *_*n*1_^*NN*^	…	*X *_*nn*_^*NN*^	*Y *_*n*_^*NA*^	*…*	*Y *_*n*_^*NN*^	*X *_*n*_^*N*^
Added value		…	…	…	…								
Total investment		*X *_1_^*A*^	…	*X *_*n*_^*A*^	…	*X *_1_^*N*^	…	*X *_*n*_^*N*^					

**Table 2:** Industry division.

Industry famous forest	Number	STTC-Rev.3 code
Agriculture, forestry, animal husbandry and sideline fishery	C1	001, 25, 34, 36, 41, 43, 57
Mining industry	C2	321, 322, 333, 342, 342, 381, 282, 283, 284, 285, 287, 288, 289
Food beverage tobacco	C3	74, 111, 112, 122, 11, 12, 16, 17, 22, 23, 24, 35, 37, 42, 45, 46, 47, 48, 54, 56, 58, 59, 61, 62, 71, 73, 75, 81, 91, 98, 411, 421, 422, 431
Textile and textile manufacturing	C4	269, 651, 652, 653, 34, 655, 36, 657, 658, 659, 841, 842, 843, 844, 845, 846, 848
Leather and leather products manufacturing	C5	611, 612, 613, 831, 851
Wood processing industry	C6	244, 245, 246, 247, 248, 633, 634, 635
Paper and printing industry	C7	251, 641, 642, 892
Coke, coal to petroleum and nuclear fuel	C8	325, 334, 335

**Table 3:** Classification of five industries.

Industry classification	
Primary and natural resources	Y1, 2
Energy industry	Y7, 22
Service industry	Y19, 22–28, 32, 34-35
Light industry	Y3–6, 10
Heavy industry	Y8, 10–18, 20

**Table 4:** Industry details.

Industry details			
Y1	Agriculture, forestry, animal husbandry, and fishery	Y17	Medical precision optical instrument
Y2	Mining and quarrying	Y18	Automobile manufacturing
Y3	Food manufacturing	Y19	Other transportation equipment
Y4	Textile industry	Y20	Other manufacturing
Y5	Wood processing industry	Y21	Water and electricity supply
Y6	Paper printing industry	Y22	Construction
Y7	Petroleum refining and chemical industry	Y23	Wholesale and retail
Y8	Chemical and pharmaceutical industry	Y24	Accommodation and catering industry
Y9	Rubber and plastic industry	Y25	Communications and transportation industry

## Data Availability

The labeled dataset used to support the findings of this study is available from the corresponding author upon request.
